The article "The Construction of Big Data Computational Intelligence System for E-Government in Cloud Computing Environment and Its Development Impact" was retracted in 2023. Reasons: signs of a paper mill; suspected computer-generated content; unreliable results or conclusions; concerns about the data.

# The Construction of Big Data Computational Intelligence System for E-Government in Cloud Computing Environment and Its Development Impact

**DOI:** 10.1155/2022/7295060

**Published:** 2022-03-24

**Authors:** Shengqing Ma, Fei Hao, Youwu Lin, Yinjing Liang

**Affiliations:** ^1^School of Economics and Management, Qinghai Normal University, Xining, Qinghai 810000, China; ^2^School of Computer Science, Shaanxi Normal University, Xi'an, Shaanxi 710119, China; ^3^School of Mathematics and Computing Science, Guilin University of Electronic Technology, Guilin, Guangxi 541004, China; ^4^College of Marxism, Taiyuan University of Technology, Taiyuan, Shanxi 030600, China

## Abstract

The traditional E-government big data system fills and classifies algorithms with low accuracy and poor work efficiency. With the development and wide application of big data, the internet of things, and other technologies, the integration of information resources has become the key to information construction. In the process of information resource integration, there are still outstanding problems such as incomplete government information resource system, different standards of government information resource management system construction, and serious threats to network and information security. In order to solve this problem, a new E-government big data system filling and classification algorithm is studied in the cloud computing environment; E-government big data filling is carried out on the basis of complete compatibility theory; and the E-government big data computing intelligence system in the cloud computing environment is constructed and its development impact, so as to parallelize the data, classify the data through decision trees, and realize incremental update decision forest parallelization processing. To verify the effectiveness of the method, comparative experiments are set, and the results demonstrate that experiment one is randomly built into the classification model, and according to the decision forest algorithm, the optimal number of decision trees is 24.

## 1. Introduction

With the rapid development and widespread use of big data technology, people are increasingly optimistic about the future of big data [1]. In particular, the increasing volume of data in recent years has made it difficult for existing software to process it effectively, and the quality of big data makes “big data” technology stand out from the crowd. Big Data can help people extract valid information from large amounts of data quickly and help them get answers quickly [2]. McKinsey & Company, the first to coin the phrase “big data era,” has pointed out that data is everywhere and that its value today is not just information but also a factor of production. Deeper mining and organization of data can help people obtain data products. “Big data strategy” is also on the agenda with the widespread use of big data [3]. Big data technology can be used to collect, process, and handle large amounts of data and analyze them from a professional perspective. People can obtain valuable information.

The article "The Construction of Big Data Computational Intelligence System for E-Government in Cloud Computing Environment and Its Development Impact" was retracted in 2023. Reasons: signs of a paper mill; suspected computer-generated content; unreliable results or conclusions; concerns about the data.

The use of big data technology for the construction of government information resources integration began to involve the construction of the platform, the construction of the information security system, the promotion of big data awareness, and other aspects, not a quick fix [4]. Big datum is more active in the construction of platforms, and many local governments are building local big data platforms to integrate government information resources across platforms and data types through the construction of big data platforms [5]. Big data platforms can help us gather a large amount of data and analyze and evaluate these data [6]. We can understand the meaning behind these data. If we just look at the data, it is sometimes difficult to get useful information from it. Big data platforms help managers change the way they used to make decisions based on personal experience and personal knowledge, and through the analysis of data, decisions can be justified, and decision-makers can quickly understand the situation through data analysis [7].

Although big data technology is widely used in the integration of government information resources, there is still a lack of big data awareness in the concrete implementation [8]. Although claiming to use big data to solve problems, the original approach is still used in problem-solving. All these show a lack of awareness of big data and the need to fundamentally understand the importance of big data and the position it occupies in the process of government transformation. At the same time, data security has become an inescapable issue as we make extensive use of data today [9, 10]. The nature of big data allows it to respond quickly to government information, which is why it is so effective in advancing the integration of government information resources so quickly.

The amount of data in the data centre is huge; therefore, it is necessary to improve the efficiency of data processing. Therefore, the paper proposes an E-government big data system filling algorithm to address the problem of data loss that occurs when the government uses the E-government big data system, which solves the problem of missing data, and proposes a parallel optimization of E-government big data system filling based on the cloud computing environment, which greatly improves the efficiency of filling missing data [11]. A new classification model for E-government big data systems in a cloud computing environment is constructed in the paper. By using a decision forest algorithm to classify and process huge data and incremental update processing of the decision forest algorithm, the big data system can continuously change its model according to the continuous change of data, and finally, the parallel optimization of the algorithm is carried out, which makes the processing efficiency greatly improved [12]. The results of the experimental demonstration of the proposed method show that the E-government big data system in the cloud computing environment proposed in the paper has great advantages over the algorithms used in the traditional way.

The article "The Construction of Big Data Computational Intelligence System for E-Government in Cloud Computing Environment and Its Development Impact" was retracted in 2023. Reasons: signs of a paper mill; suspected computer-generated content; unreliable results or conclusions; concerns about the data.

## 2. Related Work

The application of big data in government information integration will promote efficient use and innovation of government information [13]. In conclusion, big data are data that transcend traditional data analysis and processing capabilities and are difficult to apply to existing database architectures, and traditional software tools are difficult to access, store, manage and analyze, and thus, new tools and processing methods should be adopted. At the same time, big data are changing the traditional sampling data to all data by changing the precise directional hybrid transformations required from the previous precision to hybridity, more analysis, and speculation about the trend of things rather than the previous focus on cause and effect.

Yan et al. [14] propose that digital information resources have changed in the big data environment and discuss the three directions of cloud-based information resource services and active innovative service models based on relational networks and Web 2.0. Wei [15] takes the concept and characteristics of cloud computing as an entry point and uses a two-layer perspective to build a top-level design model for information technology. Long et al. [16] think in the direction of using multiple subjects to develop government information resources; propose three new paradigms of using information resources, such as the single information flow model of users, the collaborative model, and the two-way information flow model of users; and explains that the collaborative model of developing and using community information resources has obvious advantages. Fu and Sun [17] discuss the concept of government information resource exploitation and development and propose different positions of public interest and commercial exploitation of government information resource development models according to the development and exploitation models of European and American governments, aiming to give suggestions on the problems and current situation of government information resource development and exploitation [18, 19]. Through the analysis of the development of information resources in China, the importance of knowledge management in the management of government information resources is elaborated, and the strategy of using knowledge management in the development and utilization of government information resources is proposed. Through a survey of 300 valid questionnaires on the impact of big data on community management and influence, the majority of people affirmed that big data can help the government improve scientific and rational decision-making [20, 21].

The article "The Construction of Big Data Computational Intelligence System for E-Government in Cloud Computing Environment and Its Development Impact" was retracted in 2023. Reasons: signs of a paper mill; suspected computer-generated content; unreliable results or conclusions; concerns about the data.

Literature [22] put forward the idea of further refinement and transformation of China's Comprehensive E-government Thesaurus, providing suggestions for further improvement and changes to the Comprehensive E-government Thesaurus. Hernandez-Marin et al. [23] propose the idea of further refinement of China's Comprehensive E-government Thesaurus. Literature [24] explained the two major government metadata standards DC__government and GILS in the world today from a holistic perspective and put forward suggestions for building a government metadata architecture in China. There are also some scholars who have applied theme maps to the integration of government information resources, providing new methods and approaches to the integration of many E-government information resources, such as [25] and others who have applied theme maps to government portals for analysis and research. Through the analysis and consideration of methods and technologies related to E-government information resources, we can easily see that the current research on the integration of government information resources in China is mostly in the theoretical aspect, while there are not many applications for specific government information resources integration research. In the face of the vast amount of information resources, we should study and explore in depth, using the emerging big data, cloud computing, and internet of things technology to find effective solutions.

## 3. Government Information Resources Integration Solutions

In the big data environment, big data and cloud computing technology bring new development opportunities to the integration of government information resources. Big data technology can effectively solve the problems of departmental compartmentalization and unequal information standards in the previous E-government era, and big data technology will undoubtedly promote the development of China's government management in the direction of intelligence. Our government has been actively planning the construction of a big data platform for government information. By analyzing the current situation and problems of government information resource integration and construction under the big data environment, we propose complete solutions to the problems existing in government information resource integration [26].

The article "The Construction of Big Data Computational Intelligence System for E-Government in Cloud Computing Environment and Its Development Impact" was retracted in 2023. Reasons: signs of a paper mill; suspected computer-generated content; unreliable results or conclusions; concerns about the data.

### 3.1. Principles of Integration of Government Information Resources

As shown in Figure 1, in the process of integration of government information resources, the government should actively play the leading role of policy guidance, organization and collaboration, standardization, and control of the overall situation to promote the further development of government information resources. At the same time, the integration of government information resources should not only meet the requirements of government departments for the integration of information resources but also meet the requirements of the general public for government information. We should put the principle of serving the people into practice, think what the people think, and sense the urgency of the people. Starting with the most urgent need of the people, we should actively prioritize the integration of government affairs, transportation, and medical services, which are the most popular areas, and gradually realize the full implementation and development of the integration of government information resources [27].

In turn, it eliminates the problem of information silos, thus realizing the integration and sharing of information resources across industries, fields, and shutters and enhancing the effectiveness of government information utilization and the scientific nature of decision-making. Government information can hardly play its proper role if it is only within the government, and there is the use of enterprises to fully explore its potential value but also to further stimulate the demand of potential consumers, which in turn promotes the opening and use of information. While promoting the development of information technology, it also leads to the development of new information industries and the creation of new economic growth points, making the interconnection of information more fluid [28].

### 3.2. Government Information Integration Framework and Content Building

The big data platform for government affairs is mainly built by six parts, with the standard specification and information security system as the guarantee and the corresponding platform construction for infrastructure as well as database system and application system as shown in Figure 2.

The public information big data system is based on the collection of information, data exchange, and integration of information to the final information service, with the integration of the following main parts, as shown in Figure 3.

The article "The Construction of Big Data Computational Intelligence System for E-Government in Cloud Computing Environment and Its Development Impact" was retracted in 2023. Reasons: signs of a paper mill; suspected computer-generated content; unreliable results or conclusions; concerns about the data.

The integration of government information resources is carried out at three main levels, based on standard specifications and secure application systems for infrastructure, systems, and related applications.

## 4. Big Data System for E-Government in Cloud Computing Environment

In today's cloud computing environment and big data era, the scale of energy consumption big data in the big data centre of E-government is very large; often data collection information is lost during equipment failure, unexpected power failure, and other unstable factors, resulting in the lack of data information and damage, causing losses; the previous way to solve this difficulty usually uses rough set theory. However, a rough set theory can only handle small batches of data, and the processing is very tedious [29]. Based on this, a complete compatibility theory extended from the theory of compatibility relations is proposed in this paper, and based on this theory, an algorithm for filling the E-government big data system is proposed to solve the problem of missing attribute values of data in E-government data centres [24]. The management architecture of the E-government big data system is shown in Figure 4.

As can be seen in Figure 4, the entire management architecture contains a data centre, cluster monitoring module, and sensors. The raw data set is obtained using cluster monitoring to obtain the raw data set that can be used for operation and provide data for later data filing and classification. The paper proposes an E-government big data filling algorithm based on the theory of completeness and compatibility as a solution to the problem of missing data in E-government data centres. The main process of the process is to discrete the attribute values of the data, interrupt their continuity, screen out the missing data information for separation processing, arrange the attribute values for processing, then perform inverted indexing processing, and then detect whether the missing data are perfect-compatible class data; if it is perfect compatible data, the principle of minimum value is applied, and the corresponding decision attribute generated by the attribute of the corresponding condition is used to fill the missing data. If the missing data are incomplete compatibility data, the attribute value with the highest frequency of the missing attribute is used to fill the missing attribute [25].

In the process of filling in missing data, the data set is decomposed by clustering using the double clustering method, and the data set is divided into multiple data clusters with different characteristics according to the differences in the data characteristics, using the clustering idea that the smaller the average residual within the data cluster, the higher the similarity of the data within the cluster. The problem of solving the minimum average residual of the data clusters is transformed into a quadratic form, and the missing data values are solved using the idea of quadratic minima. The specific algorithm is as follows.

The article "The Construction of Big Data Computational Intelligence System for E-Government in Cloud Computing Environment and Its Development Impact" was retracted in 2023. Reasons: signs of a paper mill; suspected computer-generated content; unreliable results or conclusions; concerns about the data.

Let *B* be the data set, *C* be the corresponding set of expression attributes, and *a*_*ij*_ be the data elements in the multidimensional data expression matrix *D*. Let *I* and *J* denote the subsets of *B* and *C*, respectively; then the average residuals of *I* and *J* for the specified submatrix *A*_*ij*_ are calculated as follows:

(1) $$\begin{array}{c} Z\left(I,J\right)=\frac{1}{\left|I||J\right|}\sum_{i\in I,j\in J}a_{ij}\left(a_{ij}-a_{lj}-a_{iJ}+a_{IJ}\right), \end{array}$$

where *a*_*ij*_ is the mean of row *i* of the submatrix, *a*_*iJ*_ is the mean of column *j* of the submatrix, and *a*_*IJ*_ is the mean of the submatrix. When submatrix *A*_*ij*_ satisfies *Z* (*I*, *J*) ≤ *δ* (*δ* is the fitted value) and 0 ≤ *δ*, the smaller the value of *δ*, the more similar the data within the corresponding submatrix is. For a bicluster matrix *S* containing only one missing data *x*, assume that the total number of rows and columns of *S* are *m* and *n*, respectively; the rows and columns of the missing data are *p* and *q*, respectively; the sum of all data in *S* except the missing data is SUM; the values of *p* are (1, 2,…, *p* − 1, *p* + 1,…, *n*) [12]; and *q* takes values in the range (1, 2,…, *q* − 1, *q* + 1,…, *n*), and the average residual of the matrix of data clusters is given by

(2) $$\begin{array}{c} Z\left(m,n\right)=\frac{1}{mn}\sum_{i=1}^{m}\sum_{j=1}^{n}Z_{ij}, \end{array}$$

where

(3) $$\begin{array}{c} Z_{ij}={\left(a_{ij}-a_{Ij}-a_{iJ}+a_{IJ}\right)}^{2},\\ a_{ij}=\frac{1}{mn}\sum_{i=1}^{m}\sum_{j=1}^{n}a_{ij}=\frac{1}{mn}\left(x+\text{SUM}\right). \end{array}$$

Let ${\bar{A}}_{p}$ and ${\bar{B}}_{p}$ denote the average of all data in row *i* and column *j* of *S*, respectively, and *A*_*p*_ and *B*_*p*_ denote the average of row *p* and column *q* containing the missing data, respectively; then its calculation formula is

(4) $$\begin{array}{c} \left\{\begin{array}{c} A_{p}={\bar{A}}_{p}+\frac{x}{n},\\ B_{p}={\bar{B}}_{p}+\frac{x}{m}. \end{array}\right. \end{array}$$

According to the previous equation, when *i* = *p* and *j* = *q*, we get

(5) $$\begin{array}{c} Z_{ij}=\left(x-\bar{A_{p}}-\frac{x}{n}-\bar{B_{p}}-\frac{x}{m}\right)+\frac{{\left(x+\text{SUM}\right)}^{2}}{mn}, \end{array}$$

where *x* is the missing data, and then its quadratic function is calculated as follows:

(6) $$\begin{array}{c} Z_{ij}=c_{ij2}x^{2}+c_{ij1}x+c_{ij0}, \end{array}$$

where *c*_*ij*2_, *c*_*ij*1_, and *c*_*ij*0_ are constants.

The article "The Construction of Big Data Computational Intelligence System for E-Government in Cloud Computing Environment and Its Development Impact" was retracted in 2023. Reasons: signs of a paper mill; suspected computer-generated content; unreliable results or conclusions; concerns about the data.

The minimum value of *Z* (*m*, *n*) can be calculated by combining the nature of the quadratic function of the characteristics of the minimum value. When *Z* (*m*, *n*) is the smallest, the degree of similarity between the data is the highest, and the formula for the missing data *x* is

(7) $$\begin{array}{c} x=\frac{1}{\left(m-1\right)\left(n-1\right)}\sum_{i=U}\sum_{j=V}a_{ij}. \end{array}$$

Based on this, the filling of missing data is completed. The data that need to be processed by the E-government big data system are very large, so the proposed E-government big data system filling algorithm needs to be parallel optimized to improve efficiency. In this way, the operational efficiency of the filling algorithm for E-government big data systems can be significantly improved.

## 5. Experiment

In order to verify the effectiveness of the proposed algorithm for filling and classifying E-government big data systems based on a cloud computing environment, experimental analysis is conducted to verify.

### 5.1. Experimental Setup

In this paper, five standardized data sets, namely Abalone, CMC, Nursery, Abalone, and Yeast, were selected from the UCI machine learning database and saved as ARFF files for system testing. Basic information of the UCI data sets used is shown in Table 1.

The experiment uses distributed cloud computing on the HAD platform, with 1 high-performance PC as the master node and 19 regular PCs as slave nodes, as shown in Table 2.

In addition, the experiment will use the CloudSim simulator as the main platform for testing the filling and classification system of the E-government big data system. CloudSim will be installed, initialized, and then simulated to output the required data for testing. Data simulation flow is shown in Figure 5.

Simulation experiments can be carried out based on the above process.

### 5.2. Experimental Indicators

The experimental metrics for this experiment are divided into two parts: fill accuracy and classification accuracy.

#### 5.2.1. Fill Accuracy

Since the missing data to be processed have a certain degree of dispersion and continuity, the determination of the filling accuracy requires a combination of both cases. In the case of dispersion, the true value of the filled value is judged to be the same as the value before replacement, and if the true value is the same, then the filling is considered correct. The specific calculation formula is as follows:

(8) $$\begin{array}{c} P=\frac{\left(t_{i}+\sum_{j\in N}ag_{j}\left(\left|u_{r}-u\right|-\lambda \sqrt{S_{j}}\right)\right.}{n_{i}}, \end{array}$$

where *t*_*i*_ denotes the length of time taken to fill; *a* denotes the number of fills; *g*_*j*_ denotes the missing data finding strength factor; *u*_*r*_ and *u* denote the overall system data size before and after filling, respectively; *λ* denotes the variance; *S*_*j*_ denotes the margin of error between the filled and true values; *n*_*i*_ denotes the size of the data to be filled; and *N* denotes the set of E-government data.

The article "The Construction of Big Data Computational Intelligence System for E-Government in Cloud Computing Environment and Its Development Impact" was retracted in 2023. Reasons: signs of a paper mill; suspected computer-generated content; unreliable results or conclusions; concerns about the data.

#### 5.2.2. Classification Accuracy

The classification accuracy is a very important indicator in the evaluation of the classification effect and is calculated as follows:

(9) $$\begin{array}{c} L=\frac{\sum_{i=1}b_{i}}{N_{a}}, \end{array}$$

where *b*_*i*_ is the number of exact classifications and *N*_*a*_ is the total number of target classifications.

### 5.3. Experimental Analysis

In order to make the experiment more scientific and reasonable, the data set FX in the random function is used to select attribute values in the paper, and data sets with different missing rates are obtained. The traditional ways of filling missing values are the random forest algorithm MEAN method, the discrete random forest method FE method, and the weakly correlated random forest method ERS method, so this experiment combines the above three traditional methods with the cloud computing environment proposed in the paper for the E-government big data system The results are shown in Figure 6.

From the experimental results, it can be concluded that compared with the four methods, the proposed method of filling the big data system of E-government in the cloud computing environment makes full use of the information in the data set and significantly improves the accuracy rate, and the larger the amount of data, the more obvious the improvement is, compared with other methods; the proposed method in the paper has great advantages in quality and speed.

This experiment consists of two parts: the first part mainly records the changes in the number of decision forests in different datasets, establishes the change relationship between the classification model and time on the basis of this data, and establishes the change in the number of nodes in the classification model through this model. The analysis of the above data finally determines the relationship between the number of decision trees and time efficiency, as well as the impact on space efficiency and classification effect. In the second part, take the experimental results of the first part T and analyze the classification by comparing the classification of different data sets. This experiment proposes that the data sets filled by experiment one are randomly built into the classification model, and according to the decision forest algorithm, the optimal number of decision trees is 24, and 6/12/18/24/30/ decision trees are built in the established classification model. Each group was tested 10 times, and the average of the results was taken as the final result. The results of the first part of the experiment are shown in Figure 7.

The article "The Construction of Big Data Computational Intelligence System for E-Government in Cloud Computing Environment and Its Development Impact" was retracted in 2023. Reasons: signs of a paper mill; suspected computer-generated content; unreliable results or conclusions; concerns about the data.

Figure 7 shows the variation of time versus the number of decision trees. From Figure 7, we can see that the number of decision trees generated by the decision forest is less than 24 in the initial period, but as the number of decision trees increases, the time gradually becomes stable, and when the number of decision trees exceeds 30, the time starts to rise.

In Figure 8, it can be concluded that the number of decision forest nodes is proportional to the number of decision trees. From Figure 8, it can be found that the classification accuracy is proportional to the number of decision trees when the number of decision trees is less than 24, and the classification accuracy is inversely proportional to the number of decision trees when the number of decision trees is more than 24. This is due to the fact that the number of decisions is too many and the decision forest algorithm happens to have too many fits when performing the fitting; therefore, the number of decision trees is at the equilibrium point of classification efficiency when the number of decision trees is 24, and the second the results of the partial experiment are shown in Table 3.

As can be seen from Table 3, the proposed algorithm is far superior to the traditional random forest algorithm, discrete random forest algorithm, and weakly correlated random forest algorithm in terms of accuracy and reasonableness than the latter three. This is due to the fact that the method in the paper 8 takes into account the characteristics of E-government big data such as a large amount of information and wide data dimension and adopts the decision forest classification algorithm to provide a more refined decision strategy for the processing and analysis of the data while maintaining the updated state of the data through reconstruction processing instead of the tagged decision tree, in order to improve the accuracy of E-government big data classification.

## 6. Conclusions

In recent years, the development of cloud computing technology has become more and more mature and has a very important economic position in the development of the global industry. If cloud computing technology is applied to E-government big data systems, it has a very bright future, and the paper proposes a filling algorithm for E-government big data system based on cloud computing environment according to the problem of data loss that occurs when the government uses E-government big data centre system. The security and integrity of E-government data are ensured to avoid data missing. On the basis of this algorithm, a parallel optimization for filling E-government big data system in a cloud computing environment is proposed to further improve the efficiency of filling missing data; a decision forest algorithm based on discrete weak correlation is proposed, aiming at the parallel classification of E-government data for enhancing the processing capability of E-government data centres for data information; the paper further proposes an incremental update of the decision forest algorithm according to the decision forest algorithm; the optimal number of decision trees is 24.

The article "The Construction of Big Data Computational Intelligence System for E-Government in Cloud Computing Environment and Its Development Impact" was retracted in 2023. Reasons: signs of a paper mill; suspected computer-generated content; unreliable results or conclusions; concerns about the data.

## Figures and Tables

**Figure 1:** Principles of government information resource integration.

**Figure 2:** Big data platform system for government services.

**Figure 3:** Big data system for public information.

**Figure 4:** E-government big data system management architecture.

**Figure 5:** Simulation flow.

**Figure 6:** Comparison of the accuracy of filling in missing data sets.

**Figure 7:** Plot of time versus number of decision trees.

**Figure 8:** Number of nodes versus number of decision trees.

**Table 1:** Contents of the UCI data set.

Serial number	Data set	Number of samples	Attribute	Catalogue
1	Abalone	4,045	8	4
2	CMC	1,276	8	3
3	Nursery	11,298	8	3
4	Abalone	4,065	9	5
5	Yeast	1,439	6	4

**Table 2:** HAD platform PC configuration table.

Name	High-performance PC	Ordinary PC
CPU processor	I5-2620M	I5-2260M
Memory (GB)	8	4
Hard disk (GB)	1,024	512
Operating system	WIN7	WIN7
Operating environment	HAD-1.11	HAD-1.11

**Table 3:** Comparison of the classification accuracy of the four algorithms (%).

Number of iterations	Traditional random forest algorithm	Discrete stochastic forest algorithm	Weakly correlated random forest algorithm	Algorithm in this paper
1	78.23	76.75	80.23	95.25
2	78.64	78.47	79.45	98.34
3	86.74	80.32	81.26	94.33
4	69.04	74.85	80.54	95.25
5	71.65	79.42	83.69	96.22
6	80.59	75.73	80.83	94.34
7	75.29	76.39	79.51	96.36
8	75.84	77.54	78.84	94.86

## Data Availability

The data sets used during the current study are available from the corresponding author on reasonable request.
